# Therapeutic effect and potential mechanism of pioglitazone in rats with severe acute pancreatitis

This article has been retracted.

**DOI:** 10.1590/1414-431X20176812

**Published:** 2017-12-11

**Authors:** Wang Hai, Xu Ping, Yang Zhi-wen, Zhang Chun

**Affiliations:** 1 Department of Shanghai East Hospital, Tongji University, Shanghai, China; 2 Shanghai Songjiang Hospital, Nanjing Medical University, Nanjing, China; 3 Department of Gastroenterology, Songjiang Hospital Affiliated Shanghai First People’s Hospital, Shanghai Jiao Tong University, Shanghai, China

**Keywords:** Caspase recruitment domain-containing protein 9, Pioglitazone, Severe acute pancreatitis

## Abstract

Caspase recruitment domain-containing protein 9 (Card9) is located upstream of the nuclear factor kappa B (NF-κB) and p38 mitogen-activated protein kinase (MAPK) inflammatory pathways. This study investigated the therapeutic effect and potential mechanism of pioglitazone in rats with severe acute pancreatitis (SAP). SAP was induced by a retrograde infusion of 5.0% sodium taurocholate into the biliopancreatic duct of Sprague Dawley rats (n=54), which were then treated with pioglitazone. Blood and pancreatic tissues were harvested at 3, 6, and 12 h after SAP induction. Pancreatic pathological damage was evaluated by hematoxylin and eosin staining. Serum amylase, serum pro-inflammatory cytokines, and pancreatic myeloperoxidase (MPO) activities were determined by enzyme-linked immunosorbent assay. The expression of Card9 mRNA and protein in pancreatic tissues was detected by real-time polymerase chain reaction and western blotting. Pioglitazone had a therapeutic effect in treating rats with SAP by decreasing the level of amylase activity, ameliorating pancreatic histological damage, decreasing serum pro-inflammatory cytokine levels and tissue MPO activity, and downregulating the expression of NF-κB, p38MAPK, and Card9 mRNAs and proteins (P<0.05). The present study demonstrated that the inhibition of Card9 expression could reduce the severity of SAP. Card9 has a role in the pathogenic mechanism of SAP.

## Introduction

Acute pancreatitis (AP) is a frequent gastrointestinal emergency with high morbidity and mortality. It has been reported that approximately 25% of patients with AP develop severe acute pancreatitis (SAP) with a high mortality rate of approximately 30% (1,2). To date, the exact mechanisms of this disease have not been completely established.

Caspase recruitment domain–containing protein 9 (Card9) was recently identified as an adapter protein for host protection, and is located upstream of the nuclear transcription factor (NF-κB) and p38 mitogen-activated protein kinase (MAPK) inflammatory pathways. Card9 protein is highly expressed in macrophages and functions in many infectious diseases by regulating inflammatory signaling pathways. Card9 works with B cell lymphoma10 (Bcl10) and paracaspase, mucosa-associated lymphoid tissue lymphoma translocation protein1 (Malt1), forming a Card9–Bcl10–Malt1 complex, inducing pro-inflammatory signals via the canonical NF-κB pathway and stimulating the p38MAPK and c-June N-terminal kinase pathways (3,4). Previous studies identified the high expression of Card9 in peripheral blood mononuclear cells from patients with aseptic acute pancreatitis (5) and the potential mechanisms of therapeutic effects through siRNA silencing of the Card9 gene (6).

Pioglitazone is a special ligand of peroxisome proliferator-activated receptor-γ (PPAR-γ). It has been proved to alleviate the severity of SAP markedly, and the mechanism was most likely through the inhibition of NF-κB inflammatory pathways (7). In this study, a change in the severity of SAP was observed following treatment with pioglitazone in rats, and the change in the expression of Card9 was observed in pancreatic tissues to investigate the possible role of Card9 in the mechanisms of SAP.

## Material and Methods

### Animal grouping and preparation of the SAP rat model

Fifty-four healthy adult male Sprague Dawley rats weighing 200–250 g were obtained from the Experimental Animal Center of Shanghai Jiao Tong University [Certification of Experimental Animal: No. SYXK (Hu) 2009-0086]. The animals were housed in separate cages containing wood shavings in a temperature-controlled environment with a 12-h light-dark cycle and received food and water. All animals were allowed to acclimate for approximately 1 week. The animal experimental protocol was approved by the Ethical Committee for Animal Experiments of Shanghai Jiao Tong University, and all animal experiments agreed with the National Animal Welfare Law of China.

The rats were randomly assigned to the sham operation group (SO), SAP model group (SAP), and pioglitazone group (Pi). Each group (n=18) was further subdivided into three groups for the time points of 3, 6, and 12 h, with 6 rats in each subgroup. A midline laparotomy was performed after surgical anesthesia by an intraperitoneal injection of 4% pentobarbital. SAP was induced by a retrograde infusion of 5.0% sodium taurocholate (STC, 1 mL/kg) into the biliopancreatic duct. Thirty minutes before and after establishing the SAP model, the rats in the pioglitazone group were injected intraperitoneally with pioglitazone (50 mg/kg). In the sham group, the duodenum and pancreas were moved around, and no infusion was administered. In all groups, pancreatic tissue and blood samples were obtained at 3, 6, and 12 h after biliopancreatic duct infusion of STC. Serum was obtained and preserved at –80°C for enzyme-linked immunosorbent assay (ELISA) and other assays. Pancreatic tissue samples were obtained, and part of the tissue samples was immediately frozen and kept at –80°C for myeloperoxidase (MPO), real-time polymerase chain reaction (PCR), and western blot. The remaining pancreatic specimens were immediately fixed in 10% formaldehyde for hematoxylin and eosin (HE) examination.

### Histopathological examination

The pancreatic tissue specimens from each rat were prepared and fixed in 10% neutral-buffered formaldehyde, embedded in paraffin, cut into 4-µm thick sections, and stained with HE. Each section was evaluated by a pathologist who was blind to the study, and the following variables were determined: edema, acinar necrosis, inflammation, hemorrhage, and perivascular infiltrate. The sections were evaluated for severity of pancreatitis using a scale of 0–4 (normal to severe) as previously described by Schmidt et al. (8). The pathological scores were obtained by adding these different scores.

### Serum amylase and inflammatory cytokines

At each time point, blood was collected to measure amylase activity using an automated biochemistry analyzer. The levels of inflammatory cytokines, tumor necrosis factor (TNF)-α, interleukin (IL)-1β, and IL-6 in serum, were analyzed using ELISA kits (eBioscience, Austria) following the manufacturer's instructions.

### Pancreatic MPO activity

The pancreatic samples were thawed and homogenized in ice-cold buffer, pH 7.4. The homogenates were centrifuged at 5000 *g* for 10 min at 4°C and then the resulting pellet was resuspended in 50 mM PBS, pH 6.0 (eBioscience, Austria). The suspension was subjected to freezing and thawing for 2 h and then disrupted by sonication for 40 s. Then, the sample was centrifuged at 1000 *g* for 5 min at 4°C, and the supernatant was used for the MPO assay following the manufacturer's instructions.

### Real-time PCR

The expression of NF-κB, p38MAPK, and Card9 mRNAs in pancreatic tissue was analyzed by real-time PCR. The primer sequences for glyceraldehyde 3-phosphate dehydrogenase were as follows: forward 5′-GTCGGTGTGAACGGATTTG-3′ and reverse 5′-TCCCATTCTCAGCCTTGAC-3′. The primer sequences for NF-κB were as follows: forward 5′-CAT ACG CTG ACC CTA GCC TG-3′ and reverse 5′-TTT CTT CAA TCC GGT GGC GA-3′. The primer sequences for p38MAPK were as follows: forward 5′-TAG ACG AAT GGA AGA GCC TGA-3′ and reverse 5′-ACA GTG AAG TGG GAT GGA CAG-3′. The primer sequences for Card9 were as follows: forward 5′-TCTTTCGCAGACCCATGACA-3′ and reverse 5′-GTCGTATTCCCGTGATCCCC-3′ (Sangon Biotech, China). Total RNA was extracted from each tissue sample using TRIzol reagent (Invitrogen, USA) according to the manufacturer's instructions and subjected to reverse transcription using the reagent kit (Takara, Japan). The mixture was allowed to react in a DNA thermal cycler (Roche, USA). The relative mRNA levels were normalized to the mRNA level of glyceraldehyde-3-phosphate dehydrogenase (GAPDH). The incubation and thermal cycling conditions were as follows: denaturation at 95°C, annealing and extension at 60°C, each step for 30 s and for 40 cycles. The fold change in the expression level of each mRNA relative to all the prepared groups was calculated using the comparative CT (2^-ΔΔCT^) method.

### Western blot

The expression of NF-κB, p38MAPK, and Card9 in the pancreas at 3, 6, and 12 h were detected by western blotting. In short, a part of the frozen samples was disposed in ice-cold lysis buffer containing protease inhibitors. Then, the protein was separated by 10% sodium dodecyl sulfate–polyacrylamide gel electrophoresis and transferred to nitrocellulose membranes. Subsequently, the membranes were blocked with 5% nonfat milk overnight at 4°C. After blocking, the membranes were incubated with primary antibodies against NF-κB, p38MAPK, Card9, p-NF-κB, p-p38MAPK, and p-Card9 (ZSGB-BIO, China) overnight and with horseradish peroxidase–conjugated secondary antibodies (ZSGB-BIO) for 1 h. The bands were obtained using an enhanced chemiluminescence western blotting detection system (Thermo, USA). β-actin was used as an internal reference for relative quantification.

### Statistical analysis

Data are reported as means±SD. All experiments were independent of each other and repeated thrice. Statistical significance was assessed by a one-way analysis of variance using SPSS 21.0 (SPSS, USA). All tests were two-tailed, and a P value <0.05 was considered statistically significant.

## Results

### Serum amylase activity

Serum amylase activity in rats at all time points is shown in Figure 1. The concentrations of serum amylase in rats with SAP were significantly higher than those in the SO group (P<0.05). However, the serum amylase level in the pioglitazone-treated group was significantly different at the three time points compared with rats with SAP (P<0.05).

**Figure 1.** Serum amylase (AMS) in each group at 3, 6, and 12 h. Data are reported as means±SD. *P<0.05 compared with the sham operation (SO) group; ^#^P<0.05 compared with the severe acute pancreatitis (SAP) group (ANOVA). P: pioglitazone group.

### Histopathological examination

Significant histological changes and pathological scores in pancreatic tissues are shown in Figures 2 and 3. Tissue edema, leukocyte infiltration, acinar cell necrosis, land hemorrhage were assessed to measure the severity of pancreatitis in all rats in each group. The SO group displayed nearly normal pancreatic structure, and the pathological scores were minimal (Figure 2A–C). Pancreatic tissue injury in rats with SAP was distinct, histological changes were obvious, and pathological scores were elevated compared with the SO group. As time increased, histological changes were aggravated, and the pathological scores were markedly elevated (Figures 2D–F and 3; P<0.05). Treatment with pioglitazone ameliorated pancreatic injury, decreased pathological scores, and attenuated the severity of SAP in rats at 3, 6, and 12 h, respectively (Figures 2G–I and 3; P<0.05, at 3, 6, and 12 h).

**Figure 2.** Histopathological examination of the pancreas (hematoxylin and eosin staining, original magnification, ×400). *A*, SO group, 3h; *B*, SO group, 6h; *C*, SO group, 12h; *D*, SAP group, 3h; *E*, SAP group, 6h; *F*, SAP group, 12h; *G*, Pi group, 3h; *H*, Pi group, 6h; *I*, Pi group, 12h. SO: sham operation group; SAP severe acute pancreatitis group, Pi: pioglitazone group.

**Figure 3.** Analysis of pathological scores for pancreatic tissues at 3, 6, and 12 h. Data are reported as means±SD.*P<0.05 compared with the sham operation (SO) group; ^#^P<0.05 compared with the severe acute pancreatitis (SAP) group (ANOVA). P: pioglitazone group.

### Inflammatory cytokine levels in sera and tissue MPO

Serum inflammatory cytokine levels were measured by ELISA, and the results suggested that SAP rats had significantly increased the expression of pro-inflammatory cytokines TNF-α, IL-1β, and IL-6 (Figure 4). In addition, the level of TNF-α in SAP rats increased and reached a peak at 6 h after pancreatitis was induced, and then gradually decreased. However, these levels were significantly changed following treatment with pioglitazone. In addition, treatment with pioglitazone reduced SAP-induced MPO activity in tissues. These results demonstrated that pioglitazone effectively attenuated pancreatic injury.

**Figure 4.** Expression of serum inflammatory cytokines, tumor necrosis factor (TNF)-α, interleukin (IL)-1β, and IL-6, was analyzed by ELISA, and pancreatic tissue myeloperoxidase (MPO) activity was detected in each group at all time points. Data are reported as means±SD. *P<0.05 compared with the sham operation (SO) group; ^#^P<0.05 compared with the severe acute pancreatitis (SAP) group (ANOVA). P: pioglitazone group.

### Expression of NF-κB, p38MAPK, and Card9 mRNAs

The expression of NF-κB, p38MAPK and Card9 mRNAs increased in pancreatic tissues of SAP rats at the three time points compared with the SO group (P<0.05). In addition, significant differences were observed between the Pi and SAP groups (P<0.05). These findings suggested that treatment with pioglitazone downregulated the expression of NF-κB, p38MAPK, and Card9 mRNAs in the pancreatic tissues of rats with SAP (Figure 5).

**Figure 5.** Measurement of Card9, NF-k and p38MAPK mRNA in each group at 3, 6, and 12 h. Data are reported as means±SD. *P<0.05 compared with the sham operation (SO) group; ^#^P<0.05 compared with the severe acute pancreatitis (SAP) group (ANOVA). Pi: pioglitazone group.

### Expression of NF-κB, p38MAPK, and Card9 proteins

A lower level of NF-κB, p38MAPK, and Card9 proteins in pancreatic tissues were found in the SO group. The levels strongly increased in the SAP group compared with the SO group. However, the expression of NF-κB, p38MAPK, and Card9 proteins in the pancreas was markedly lower in the Pi group, than that in the SAP group (Figures 6 and 7, P<0.05).

**Figure 6.** Expression of NF-κB, p38MAPK proteins at 3, 6, and 12 h was analyzed by western blotting in each group. Data are reported as means±SD. *P<0.05 compared with the sham operation (SO) group; ^#^P<0.05 compared with the severe acute pancreatitis (SAP) group (ANOVA). Pi: pioglitazone group.

**Figure 7.** Expression of Card9 proteins at 3, 6, and 12 h was analyzed by western blotting in each group. Data are reported as means±SD. *P<0.05 compared with the sham operation (SO) group; ^#^P<0.05 compared with the severe acute pancreatitis (SAP) group (ANOVA). Pi: pioglitazone group.

## Discussion

A rat model of SAP was established in this study using STC-induced pancreatitis, which has been widely used and is the most successful model of the evolution of AP (9). Tissue edema, leukocyte infiltration, acinar cell necrosis, and hemorrhage were the pathological changes observed in this model. The activation of NF-κB and p38MAPK inflammatory pathways has also been observed in this model (10,11). The pathogenic mechanisms of AP are still incompletely understood; the NF-κB and p38MAPK were confirmed as two main pathways involved in the changes in pro-inflammatory cytokines in SAP (12).

Card9 was confirmed to be an important binding protein highly expressed in myeloid cells, especially in antigen-presenting cells such as dendritic cells and macrophages (13). Card9 can mediate the NF-κB and p38MAPK inflammatory signaling pathways by directly binding to Bcl10/leukemia and Malt1 (1). As the upstream regulator of NF-κB and p38MAPK inflammatory signaling pathways, Card9 can induce macrophages to produce or release inflammatory factors and has a vital role in macrophage inflammatory activation *in vitro* (12). Card9 has recently been proposed to mediate the development of chronic intestinal inflammation (14,15). Previously, the role of overexpression of Card9 in peripheral blood mononuclear cells was discovered in patients with SAP (5). The inflammatory response in pancreatic tissue was found to be reduced by blocking the activation of NF-κB and p38MAPK via si-RNA-mediated gene knockdown of Card9 (6).

PPAR-γ has been proved to be involved in the metabolism of glucose and adipogenesis (16,17). In addition, PPAR-γ ligands have been reported to possess anti-inflammatory functions *in vitro*. For example, PPAR-γ ligands can decrease the secretion of TNF-α, IL-1β, and IL-6 in monocytes and macrophages (18), thereby alleviating the severity of SAP (7,19,20). A recent study (21) indicated that the activation of PPAR-γ led to the inhibition of Dectin-1-induced activation of the NF-κB and MAPK signaling cascades by reducing the expression of Card9. Therefore, Card9 was considered to play a vital role in the mechanism of AP, and was confirmed to be a new therapeutic target for AP with further studies. Meanwhile, Card9 may play a positive role in the treatment of SAP by pioglitazone by inhibiting the activation of the NF-κB and MAPK inflammatory signaling pathways.

In the present study, the serum level of amylase in the pioglitazone-treated group decreased more significantly than that in the SAP group. This was in accordance with the results of the histopathological examination, which also showed less inflammatory cells, edema, hemorrhage, and necrosis in pancreatic tissue in the pioglitazone-treated group. The pathological scores of pancreatic tissues in the pioglitazone group were significantly lower than those in the SAP group, demonstrating that pioglitazone effectively protected the pancreas and alleviated inflammatory reactions.

Recent findings demonstrated that as the major mediators, pro-inflammatory cytokines played a crucial role in the pathogenesis of AP (22). In addition, it was revealed that restricting the expression of pro-inflammatory cytokines reduced the severity of AP (23). The NF-κB and MAPK inflammatory signaling pathways play important roles in the pathogenesis of AP (24). The present study showed that the serum levels of TNF-α, IL-1β, and IL-6 in the SAP group were significantly higher than those in the SO group. These findings indicated that the severity of SAP was aggravated. Following treatment with pioglitazone, the secretion of pro-inflammatory cytokines TNF-α, IL-1β, and IL-6 reduced significantly.

The results showed that pioglitazone could inhibit the release of serum cytokines TNF-α, IL-1β, and IL-6 and decrease the pancreatic MPO activity, thus attenuating the severity of SAP. Furthermore, the expression of NF-κB, p38MAPK, and Card9 mRNAs in the SAP group increased continuously compared with the SO group, and the expression of NF-κB, p38MAPK, and Card9 mRNAs and proteins in the Pi group was statistically different from that in the SAP group. Indeed, the expression of Card9 in pancreatic tissues changed with the severity of SAP.

Previous studies (19,25) reported that the synthetic PPAR-γ ligand, pioglitazone, significantly attenuated the severity of SAP in rats by inhibiting the inflammatory signaling pathways. Interestingly, in the present study, pioglitazone not only reduced the expression of Card9 but also alleviated the severity of SAP. This finding was in accordance with previous studies (24), indicating that the activation of PPAR-γ led to the inhibition of activation of NF-κB and MAPK signaling pathways by reducing the expression of Card9. Therefore, it was postulated that the anti-inflammatory effect of pioglitazone in STC-induced pancreatitis might be due, in part, to the inhibition of activation of inflammation signaling pathways, and Card9 might be implicated in the pathogenesis of SAP by inhibiting the activation of NF-κB and MAPK signaling pathways.

In summary, this novel study showed that Card9 might be a new therapeutic agent for STC-induced pancreatitis in rats. Further studies are required to validate the findings.
